This article has been retracted.

# RNAi-mediated silencing of vitellogenin gene curtails oogenesis in the almond moth *Cadra cautella*

**DOI:** 10.1371/journal.pone.0245928

**Published:** 2021-02-11

**Authors:** Mureed Husain, Khawaja Ghulam Rasool, Muhammad Tufail, Waleed Saleh Alwaneen, Abdulrahman Saad Aldawood

**Affiliations:** 1 Plant Protection Department, Economic Entomology Research Unit, College of Food and Agriculture Sciences, King Saud University, Riyadh, Saudi Arabia; 2 Ghazi University, Dera Ghazi Khan, Punjab, Pakistan; 3 National Center for Agricultural Technology (NCAT), King Abdulaziz City for Science and Technology (KACST), Riyadh, Saudi Arabia; Harran University, TURKEY

## Abstract

Vitellogenins, major yolk protein precursors, play an essential role in the reproduction and spread of all oviparous species, including insects. To investigate reproductive strategies of the warehouse moth *Cadra cautella* at the molecular level, a partial transcript of the *C*. *cautella* vitellogenin (*CcVg*) gene was extended through the rapid amplification of cDNA ends PCR and sequenced. The complete *CcVg* mRNA transcript was 5,334 bp long, which encoded a protein of 1,778 amino acids, including the first 14 amino acids of the signal peptide. The deduced *CcVg* protein contained a putative cleavage site (RTRR) at the amino-terminal side, similar to several other insect species. DGQR and GI/LCG motifs were present at the *CcVg* gene C-terminus, followed by nine cysteine residues. *CcVg* harbored 131 putative phosphorylation sites, numbering 84, 19, and 28 sites for serine, threonine, and tyrosine, respectively. The transcript showed a great resemblance with other lepidopteran Vgs. *CcVg* protein analysis revealed three conserved regions: 1) vitellogenin-N domain, 2) DUF 1943 (domain of unknown function), and 3) a von Willebrand factor type D domain. Additionally, sex, stage-specific, and developmental expression profiles of the *CcVg* gene were determined through RT-PCR. The *Vg* was first expressed in 22-day-old female larvae, and its expression increased with growth. The phylogenetic analysis based on different insect Vgs revealed that the *CcVg* exhibited close ancestry with lepidopterans. The *CcVg*-based RNAi experiments were performed, and the effects were critically evaluated. The qRT-PCR results showed that *CcVg*-based dsRNA suppressed the *Vg* gene expression up to 90% at 48 h post-injection. Moreover, *CcVg*-based RNAi effects resulted in low fecundity and egg hatchability in the *CcVg*-based dsRNA-treated females. The females laid eggs, but because of insufficient yolk protein availability the eggs could not succeed to hatch. The significant difference in the fecundity and hatchability unveils the importance of *CcVg* gene silencing and confirmed that the *Vg* gene plays a key role in *C*. *cautella* reproduction and it has the potential to be used as a target for RNAi-mediated control of this warehouse pest.

## Introduction

Pests and disease have always threatened agricultural commodities throughout the farm to table process. The date palm, *Phoenix dactylifera* (Linnaeus 1753), is a primitive tree that has been cultivated worldwide, including the Arabian Peninsula [1, 2]. Dates are highly valued annual fruits that must be stored after harvesting for processing and marketing. Major postharvest loss in date fruit quantity and quality can occur because of insect infestations. Date fruits are highly nutritious and very popular foods in the Middle East [3]. Saudi Arabia grows several million date palms on an estimated 107,281 hectares of land annually, producing 1,095,158 tons of date fruit, adding more than 2 billion Saudi Riyals of revenue per year [4, 5].

Although several lepidopteran pests attack date fruits, the almond moth, (*Cadra cautella*) (Walker) (Lepidoptera: Pyralidae) is a major date fruit pest [6–8]. The *C*. *cautella* damage date fruits when the fruit is still on the tree, infest date fruits in storehouses, and can produce several generations per year under suitable environmental conditions [9]. The presence of juveniles inside dates degrades the quality, aesthetic value, which ultimately influences product marketability. Larvae cause considerable damage by feeding gregariously on stored date fruits. Larvae bore inside the fruits and remain there for the duration of the larval stage. During the last instars, larvae leave the feeding area, stop feeding, secrete silk, and look for an appropriate place to pupate. Larval stages observed at 25°C on artificial feed and Khodri date diets were 28 and 48 d long, respectively. The pupal stage remains for 8–10 days. After adult emergence, the female looks for a male to have copulation within 6–10 hours. After mating female starts egg laying within the 24 hours. The oviposition period remains almost for 4–7 days and a normal female moth can produce 300–450 eggs during her lifetime [10, 11].

Pertaining to the control of *C*. *cautella*, phosphine and methyl bromide are very good fumigants; however, they have certain limitations, and since methyl bromide was stated as an ozone layer-damaging substance, its production and usage are banned globally [12]. Phosphine stimulates resistance development in insects, and longer exposure times are required to kill pests effectively [13]. Thus, several alternative control measures have been proposed to control *C*. *cautella*, including botanical extracts [14, 15], freezing effects [16], heat treatments [17], and modified atmosphere [18–20]. However, none of these approaches have been approved as potential alternatives to methyl bromide and phosphine fumigants for C. *cautella* management. Thus, the investigation of a molecular approach is required to explore an environmentally friendly *C*. *cautella* management technique.

Reproductive proliferation among all oviparous organisms is a significant biological characteristic that builds up their population. Several important genes substantially contribute to the sustenance of developing embryos inside the ovum. Among these is the vitellogenin (*Vg*) gene, which is of prime importance and plays a key role in embryonic development and insect proliferation. The molecular characterization of the *CcVg* gene will help elucidate the reproductive mechanism, which would lead to the development of safer pest management strategies.

The *Vg* genes are highly conserved in their primary structure, encoding the major yolk protein precursor that is crucial for reproduction in all oviparous animals, including insects. The *Vg* sequences have been reported in many arthropods, including insects. Some major insect species include the silkworm, *Bombyx* mori (Linnaeus) (Lepidoptera: Bombycidae) [21], yellow fever mosquito, *Aedes aegypti* (L.) (Diptera: Culicidae) [22], American cockroach, *Periplaneta americana* (Linnaeus) (Dictyoptera: Blattidae) [23, 24], Madeira cockroach, *Leucophaea maderae* (F.) (Dictyoptera: Blattidae) [25], western honey bee, *Apis mellifera* (L.) (Hymenoptera: Apidae) [26], Japanese giant silkworm, *Saturnia japonica* (Moore) (Lepidoptera: Saturniidae) [27], cotton leafworm, *Spodoptera litura* Fabricius (Lepidoptera: Noctuidae) [28], brown planthopper, *Nilaparvata lugens* (Stål) (Hemiptera: Delphacidae) [29], bed bug, *Cimex lectularius* L. (Hemiptera: Cimicidae) [30], and beet armyworm, *Spodoptera exigua* (Hübner) (Hemiptera: Noctuidae) [31]. Unequal numbers of *Vg* genes have been described among dissimilar insect species [32–34]. In *P*. *americana* and *L*. *maderae*, two *Vg* genes from each species have been reported [23–25, 35]. The bean bug, *Plautia stali* Scott (Hemiptera: Pentatomidae), has three *Vg* genes [36], whereas *A*. *aegypti* has five *Vg* genes [22, 37].

The *Vg* gene is a precursor of vitellin (Vn) protein in oviparous organisms. Vitellin protein in *A*. *aegypti* contributes to approximately 75% of the entire yolk protein [38]. In German cockroaches, *Blattella germanica* (L.) (Dictyoptera: Blattidae), Vn constitutes 93.3% of the total yolk protein [39]. Similarly, in *P*. *americana*, the total yolk protein concentration obtained from ootheca was 88% [40]. Vitellogenins encode the major yolk protein precursor, an essential part of the developing embryo food [41, 42].

Vitellogenin is sex-, tissue-, and stage-specific; it is expressed in fat body tissues, moves into the bloodstream, is taken up by its specific receptor, named the vitellogenin receptor (VgR), through receptor-mediated endocytosis, and is internalized into the developing oocytes [41, 43–45]. The *Vg* gene’s specificity with sex, tissues, and developmental stages has been documented in several insects [23, 24, 41, 44, 46]. In the rice moth, *Corcyra cephalonica* (Stainton) (Lepidoptera: Pyralidae), the *Vg* gene was first expressed in the early larval stage at a low level but was missing in the mature larval phase, re-expressed in the early pupal stage, and was present throughout the adult stage. Interestingly, a small amount of *Vg* was also present in *C*. *cephalonica*-mated males [47].

Recent biotechnological advancements have made it possible to suppress sequence-specific gene expression through RNA interference (RNAi). There are several successful examples of silencing the function of genes of interest through RNAi at the laboratory level in many arthropod groups. For example, in the Lepidoptera, the *Vg* gene of *C*. *cephalonica* has been silenced [47], in Diptera, the transferrin gene of the tsetse fly, *Glosina morsitans morsitans*, Westwood (Diptera: Glossinidae), has been successfully silenced [48], and in Hymenoptera, the *Vg* gene of the *A*. *mellifera* has been downregulated [49]. RNAi offers several opportunities regarding insect genomics, such as the study of gene functions, improving pest control, and reducing disease [50]. The study’s goal was to sequence, characterize, and silence *CcVg* gene function through RNAi technology that might improve its management.

## Materials and methods

### *Cadra cautella* rearing

The insects were reared in the laboratory in an incubator (Steridium) at 26°C ± 1°C, 60% ± 5% RH, and a 9:15 dark: light photoperiod using an artificial diet as a rearing medium [10, 11, 51]. Various stages of insects were used in the present study. Final instar female larvae were taken from the culture and kept in 50 g plastic cups where they pupated, and upon the eclosion, abdominal tissue samples were collected from 1-day-old adult female moths that were later used to synthesize cDNA and further downstream applications *Vg* extension. For *Vg* expression analysis, different stages were collected directly from the rearing culture. For RNAi application, last instar female larvae (21-days-old) were collected from the colony, and *CcVg* dsRNA was injected.

### RNA extraction and cDNA preparation

The abdomens of newly emerged female moths (1–2 days old) were cut to extract total RNA. The quality and quantity of total RNA were measured using NanoDrop. From the extracted mRNA, 1 μg was used to synthesize an adapter-ligated double-stranded (ds) cDNA library with the help of a Marathon cDNA Amplification kit (Clontech, USA) [25, 29]. The synthesized ds cDNA library was subsequently diluted in a tricine-EDTA buffer (1:50), denatured at 94°C for 2 min, and RACE-PCR was conducted to obtain *CcVg* full-length mRNA sequences.

### Amplification and sequencing of *CcVg* gene

The partial *Vg* gene transcript obtained from next-generation sequencing of *C*. *cautella* female moth abdominal tissues was extended using gene-specific primers, *CcVg*, and the adopter primer, AP (S1 Table), through RACE-PCR [25]. The *CcVg* cDNA library was used for the RACE-PCR following previously used conditions [41]. The amplified PCR product was purified.

The purified PCR product was sequenced by Beijing Genomics Institute (BGI, China). The obtained sequences were aligned with the available *CcVg* partial sequence, and a full-length mRNA transcript of *CcVg* was obtained. Using the Basic Local Alignment Search Tool, the *CcVg* gene’s homology was checked with other insect *Vg* sequences. Finally, after confirmation, the *CcVg* transcript was submitted to NCBI, and an accession number was obtained.

### Structural comparison of *Cadra cautella* Vg and phylogenetic analysis

The ExPASy translation tool was used to translate the full-length *CcVg* gene into an amino acid sequence. The acquired *CcVg* sequences were aligned with the *Vg* sequences of other known insects, including lepidopterans, accessible at NCBI (National Center for Biotechnology Information). The Clustal W program was applied for multiple alignments and structural comparisons to make the neighbor-joining phylogenetic tree.

### Expression analysis of the *CcVg* gene

Stage- and sex-specific expression of the *CcVg* transcript was investigated by extracting total RNA from different developmental stages *C*. *cautella*, containing young larvae (10 days old), mature female/male larvae (15 and 22 days old), female/male pupae (1 and 7 days old), and adult female/male moths (1 day old) [47]. To study the temporal expression profile of *CcVg*, RNA was extracted from different developmental stages (female larvae, 22–27 days old; female pupae, 1–5 days old; and female adult, 1–5 days old) as described above. DNA contaminations were removed from the total RNAs through treatment with DNase I. One to two micrograms of DNase-treated RNAs from relevant stages and sexes were transcribed reversely to cDNA. RT-PCR was conducted with specific primers (*CcVg*-RTF and *CcVg*-RTR) using the actin gene as an internal control (S1 Table). The amplicons were separated on agarose gel (1.2%), staining was performed with ethidium bromide, and the amplified products were visually confirmed in the presence of ultraviolet light.

### RNAi target region selection and dsRNA synthesis

A unique target region of 433 bp (nucleotide position: 4125–4558) that displayed no homology with other insect Vgs was selected from the C-terminus of the *CcVg* gene transcript to silence the *CcVg* function through RNAi. The targeted sequence was amplified with RNAi primers (S1 Table), having a T-7 promoter region at the 5ʹ end. The amplified PCR products were purified as described above (S1 Fig). The amplified product was run on an agarose gel to check the RNAi target region identity and purified for sequence confirmation (S2 Fig). After the confirmation of the target region, the purified product was used to produce *CcVg*-base dsRNA for RNAi application.

The dsRNA was formed. The MEGAscript^®^ RNAi kit has been successfully used in several RNAi experiments [52–54]. A reaction of dsRNA (20 μL) was set in a standard PCR tube. The dsRNA was digested with nucleases to remove DNA and ssRNA. The dsRNA was eluted in a 100 μL solution and stored at −20°C for future use. The quality of dsRNA was measured using NanoDrop (S3 Fig) gel electrophoresis (S4 Fig).

### Silencing of *CcVg* and RNAi results validation

The *CcVg*-based dsRNA was used to knockdown the function of the *Vg* gene in *C*. *cautella* females. The RNAi experiment consisted of three biological treatment groups: a *CcVg*-dsRNA-injected group, a nuclease-free water group, and a no injection (NI) group. Moreover, for RNAi application, we used last instar female larvae (21-days-old) because from the CcVg expression studies we confirmed that during the last larval instar the *Vg* gene expression begins and continue to increase till the adult stage. Because of this reason, we selected last instar female larvae (21-days-old) and injected CcVg dsRNA.

One microgram (volume: 1 μL) of *CcVg* dsRNA was injected in a 21-day-old female larva on the lateral side of the second abdominal segment. Nuclease-free water (1 μL) was injected as a control treatment. After the injection, the larvae were placed inside the incubators under the same conditions (25°C ± 1°C and 65% ± 5% RH). All 3 groups were examined after 3 exposure intervals of 24, 48, and 72 h. There were three biological treatment groups, and each group contained three replicates, whereas each replicate was a group of three larvae. After relevant exposure times, RNA was extracted from larvae, and cDNA was synthesized to observe *Vg* transcript expression through RT-PCR, qRT-PCR, and by observing RNAi’s phenotypic effects on different biological parameters, such as ovipositional times, egg laying, and egg fertility.

RT-PCR was performed using *CcVg* specific primers, and actin was used as an internal control (S1 Table). PCR was performed using similar conditions as described for the expression study. After PCR, all the samples were run on 1% agarose gel, stained with ethidium bromide, and observed in the gel documentation system.

Furthermore, RNAi effects were assessed through a quantitative real-time PCR using *CcVg*-qRT primers using the actin gene to normalize *CcVg* expression (S1 Table). A 20 μL reaction was prepared, and PCR was performed. The normalized fold expression of the *CcVg*-dsRNA-injected group compared with nucleus-free water (NFW) and NI groups at 24, 48, and 72 h post-injection. All the biological groups contained three replicates for each exposure time. Hence, each replicate had a pool of three larvae, and there were three technical replicates. The relative expression level of *CcVg* was computed and analyzed with the 2^−ΔΔCT^ method using actin and NI control groups as normalizing groups. Note that S2 Table presents the details on all the chemicals/reagents, machines, PCR conditions, and software used in the study.

Additionally, through biological studies, *Vg* gene silencing influence was validated in RNAi-treated females. In the biological studies, the treated female larvae pupated, and when the female moths emerged, they were allowed to mate with non-treated male moths of similar age. There were five pairs in each treatment group, considering one pair as a replicate, and a completely randomized design was used. The moths started mating, and biological parameters, such as the ovipositional period, fecundity, fertility, and adult longevity, were recorded until the death of all pairs under observation.

### Statistical analysis

The real-time PCR results were quantified using the 2^−ΔΔCT^ method [55]. The quantified real-time PCR data and biological studies data for all treatment groups (NI, NFW, and *CcVg*-dsRNA-injected groups) were analyzed by performing a one-way analysis of variance using SAS program ver. 9.2 (α = 0.05) [56].

## Results

### Sequencing of *CcVg* gene transcript and structural analysis

The complete *CcVg* gene transcript was 5,334 bp, which encoded a 1,778 residue mature protein that contained all conserved structures typical of insect Vgs (GenBank, accession number: ALN38805). The protein analysis predicted the first 14 amino acid residues as a signal peptide analyzed with the signal P program. The determined *C*. *cautella Vg* protein sequence only contained one putative cleavage recognition site, RTRR (amino acids, 353–356). Furthermore, *CcVg* contains DGQR and GICG conserved motifs on amino acid positions 1,574–1,577 and 1,591–1,944. At the C-terminus, *CcVg* has seven cysteine residues. *CcVg* included three putative glycosylation sites (NXT/S) determined by the NetNGlyc program. Moreover, 131 putative phosphorylation sites, numbering 19, 28, and 84 sites for threonine, tyrosine, and serine, respectively, were identified in the *CcVg* sequence (S5 Fig).

The *CcVg* protein contained three conserved domains confirmed using the conserved domain database at NCBI. These include 1) the Vg-N domain, covering 30–732 amino acids; 2) the domain of unknown function 1943 (DUF1943), covering 764–1,035 amino acids; and 3) the Von Willebrand factor domain (VWD), located at the C-terminus, covering 1,442–1,609 amino acids (Fig 1).

**Fig 1:** Schematic representation of the *Cadra cautella* full length vitellogenin (CcVg) protein. The CcVg protein is 1,778 amino acids long. The green rectangle at the beginning of the Vg-bar represents the signal peptide (SP). The numbers in the rectangle frames represent the amino acid position of three conserved domains.

### Structural comparison and phylogenetic analysis

The *C*. *cautella Vg* sequence was aligned with other insect and lepidopteran *Vg* sequences available at NCBI. The comparison revealed that *CcVg* was closely related to that of the lepidopteran species, including 79% with Navel orangeworm, *Amyelois transitella* (Walker) (Lepidoptera: Pyralidae), followed by 60% with *Corcyra cephalonica*. Moreover, the *CcVg* C-terminus structure was compared with other lepidopteran species, and in the *CcVg* sequence, GL/ICG and DGXR motifs were conserved at the C-terminus like in other lepidopterans. The DGXR motif was positioned at 13 residues upstream of the GL/ICG motif. Additionally, in *CcVg*, six cysteine residues were present at the C-terminus, similar to that of the Vgs of other lepidopteran species (Fig 2).

**Fig 2:** Structural comparison of *Cadra cautella* Vg C-terminus with other lepidopteran members. Clustal W multiple alignment program was used. The conserved DGXR, GL/ICG motifs, and cysteine (C) residue are with bright colors.

Furthermore, the evolutionary relationship of *CcVg* was elucidated through neighbor-joining phylogenetic tree analysis based on *Vg* sequences of insects and other organisms accessible at NCBI (Fig 3). In the phylogenetic tree, related insect species were coherently grouped in clusters, reflecting the higher sequence similarity within the insect group than that of other organisms. The *CcVg* sequence was successfully grouped with other lepidopteran species and linked up on the same clade with the *Vg* of *A*. *transitella*. Phylogenetic analysis showed that insect Vgs are evolutionarily closer to the Vgs of arachnids and nematodes than vertebrates (Fig 3).

**Fig 3:** Neighbor-joining phylogenetic tree of different insect Vgs representing seven insect orders. The Clustal W and MEGA 6, a neighbor-joining tree construction program, were used. A scale of 0.2 indicate the distance (a number of amino acid substitutions per site). Species belonging to different orders are marked with different colors.

### Sex and stage-specific expression

The specific expression of the *CcVg* gene was determined through RT-PCR using gene-specific primers and actin as a control (S1 Table). The results showed that the *CcVg* began to express in female larvae (22 days old); however, there was no expression in male developmental stages (Fig 4). The abbreviations are described here for the studied developmental stages of *C*. *cautella*. L = larvae, LF = larvae female, LM = larvae male, PF = pupae female, PM = pupae male, AF = adult female, and AM = adult male.

**Fig 4:** Stage- and sex-specific expression pattern of *CcVg* and actin genes. The expression pattern was studied from different developmental stages of *Cadra cautella*, analyzed by semi-quantitative reverse transcriptase PCR. The 980 bp and 763 bp on the right side are amplified products of CcVg and actin genes, respectively. M = molecular marker, bp = base pair, d = day.

Similarly, *CcVg* expression profile was studied up to 16 days (female larvae, 22–27 days old; female pupae, 1–5 days old; and female adults, 1–5 days old). The RT-PCR results revealed that *CcVg* gene expression begins in 22-day-old female larvae, gradually increasing with time and stage of development, and maximum band intensity was observed on the first day of adult female eclosion (Fig 5). The expression profile was analyzed by semi-quantitative reverse transcriptase PCR. The amplified bands were visualized under ultraviolet light and photographed using the BioDocAnalyze gel documentation system (Biometra).

**Fig 5:** Expression profile of *CcVg* in *Cadra cautella* females. The 980 bp and 763 bp on right side are amplified products of CcVg and actin genes, respectively. M = molecular marker, bp = base pair, d = day.

### *CcVg* gene silencing and validation through qRT-PCR

The real-time PCR results showed reduced *Vg* gene expression in female larvae injected with *CcVg*-based dsRNA compared with other groups. dsRNA-injected females exhibited the downregulation of *Vg* transcript up to 52%, 90%, and 73% after 24, 48, and 72 h post-injection, respectively (Fig 6).

**Fig 6:** RNAi-mediated silencing of the *CcVg* gene. Different letters above the bars (a, b) show significant differences between the treatment groups (α = 0.05). The bars represent normalized fold expression (mean ± SE).

### RNAi validation through RT-PCR

The RT-PCR data also confirmed an apparent reduction of *CcVg* expression in *C*. *cautella* females treated with dsRNA compared with other groups. However, the actin expression pattern was parallel in all experimental groups (Fig 7). These findings unequivocally showed that *CcVg*-based RNAi is target-specific as there was no effect on housekeeping actin gene expression.

**Fig 7:** Validation of RNAi-mediated *CcVg* gene silencing through RT-PCR. Arrows on the right side indicate the amplified products of *CcVg* and *actin* genes. M = molecular marker, bp = base pair, d = day.

### *CcVg* gene silencing diminish *Cadra cautella* female reproduction

To access the effects of *CcVg* knockdown on *C*. *cautella* female reproduction, the following biological parameters were examined: 1) pre-oviposition, 2) oviposition, 3) post-oviposition periods, 4) fecundity, 5) egg hatchability, and 6) female life span (Fig 8A–8D). In the Fig 8 we presented only the significant results. The results showed a difference in the pre-oviposition period of dsRNA-treated females and other groups (Fig 8A). Similarly, a significant difference in the oviposition periods of dsRNA-treated females was observed compared with that of the other groups (Fig 8B). Moreover, statistical analyses revealed a significant difference in the total number of eggs laid per female, where dsRNA-injected females laid fewer eggs than NI- and NFW-injected females (Fig 8C). Furthermore, only 40% egg hatchability was observed in *CcVg*-dsRNA-injected females, compared with NI- and NFW-injected groups with hatchability of 87% and 88%, respectively (Fig 8D). However, post-ovipositional periods and adult female life span were not statistically different among the females in the dsRNA-injected groups and NI- and NFW-injected groups.

**Fig 8:** Effects of the *CcVg* gene knockdown on *Cadra cautella* females reproductive traits. (A–B): Pre-oviposition and oviposition periods (C–D): mean number of eggs laid per female and egg hatchability.

## Discussion

This study presents *C*. *cautella Vg* gene molecular characterization and demonstrates its expression profile and evolutionary relationships among other insect Vgs. This study also reports the potential use of *CcVg* gene silencing as a tool for *C*. *cautella* management, a serious pest of date fruits. A recent molecular study proved that the major yolk protein precursors are well-preserved among different insect taxa, except in some differences during the post-translational modification process [32–34, 46]. The molecular weight of the *CcVg* protein was 200.33 kDa, predicted through ExPASy tools, which is nearly in the range of other insect Vgs, including those of lepidopterans [28, 47]. Similar to other insect Vgs, the *CcVg* contains Vg-N, DUF1943, and VWD conserved domains. The Vg-N domain may participate in lipid transportation [57], whereas the VWD domain contributes to fertilization, but the DUF1943 domain function remains unknown [58].

In most insects, *vg* precursors are post-translationally modified and cleaved proteolytically at a specific cleavage site (rxxr) into different subunits by enzyme-like dibasic endoproteases [59, 60]. The *ccvg* exhibited a cleavage motif of “rtrr” conserved at the n-terminus, where the *ccvg* protein possibly cleaves during the post-translational modification process into a small subunit (40.22 kda) and a large subunit (160.11 kda). The presence of the single cleavage site in the *vg* protein has already been reported from other lepidopteran species such as the gypsy moth, *lymentria disper* L. (Lepidoptera: Lymantriidae) [61]. The cleavage of *CcVg* at the N-terminus is not surprising because it is a common feature reported from many insect species [33, 62, 63], except the *Vg* of *L*. *disper*, where the *Vg* cleaved at the C-terminus and the C-terminus subunit is larger than that of the N-terminus [61]. However, in some lepidopterans, such as the wild silkworm, *Antheraea pernyi* (Guérin- Méneville) (Lepidoptera: Saturniidae), no cleavage site has been observed [64]. The cleavage of *Vg* molecules and post-translational modification also enable it to carry nutrients, such as carbohydrates, lipids, and sulfates from the hemolymph to developing oocytes in the ovary [32, 65].

The presence of the polyserine region in insect Vgs is a common characteristic. Usually, in most insect Vgs, polyserine clusters are present on both sides of cleavage consensus RXXR. Similar to most insect Vgs, polyserine clusters surround the *CcVg* cleavage site, and it indicates the structural similarity of *CcVg* with known Vgs of other insect species including, *A*. *pernyi* [64]; *P*. *americana* [24]; *L*. *maderae* [25]; Indian moon moth, *Actias selene* Hubner (Lepidoptera: Saturniidae) [66]; and *C*. *cephalonica* [47]. However, the absence of polyserine tracts has been reported in some insect species, including lepidopterans, such as *L*. *disper* [61], *S*. *litura* [28], and coleopterans, such as the red palm weevil, *Rhynchophorus ferrugineus* (Olivier) (Coleoptera: Dryopthoridae) [67].

Moreover, the existence of some other remarkable characteristics such as conserved GL/ICG motifs and cysteine residues are similar to those that exist in other insect Vgs, including the lepidopterans [21, 23, 28, 47, 53, 63, 68]. In the *CcVg* protein sequence, the DGQR was positioned at 13 residues upstream of the GI/LCG motif that is conserved in almost all lepidopteran Vgs [47, 64]. Additionally, *CcVg* protein sequence is highly phosphorylated, comparable with several other insect species, including cotton boll weevil, *Anthonomus grandis* Boh. (Coleoptera: Curculionidae) [53], chrysomelid beetle, *Octodonta nipae* (Maulik) (Coleoptera: Chrysomelidae) [68], and *R*. *ferrugineus* [67]. By contrast, the *Vg* of *C*. *cephalonica* has 127 phosphorylation sites, and all of them were the serine residue, whereas threonine (T) and tyrosine (Y) were absent [47].

The The phylogenetic analysis results revealed that *CcVg* was placed within a clade of the order Lepidoptera and showed close ancestry relationships with the *Vg* of *A*. *transitella* and *C*. *cephalonica*. The neighbor-joining tree based on 23 *Vg* sequences of different lepidopteran insect confirmed the phylogenetic relationship of *CcVg* at the molecular level.

In *C*. *cautella*, the *Vg* gene specifically starts expressing in 22-day-old late female larvae. The expression was witnessed throughout the female pupa and adult stage. By contrast, no expression was observed in male samples, which supports that *Vg* gene expression is sex- and stage-specific as described previously in several insect species [23, 25, 28, 29, 47, 67, 69]. The *CcVg* gene expression gradually increased with time and stage development and peaked on the first day of female eclosion. In most of the lepidopteran species, *Vg* gene expression begins during the immature stage. For example, *Vg* mRNA transcripts were first recorded at 6- and 1-day-old female pupae in *S*. *litura* and *A*. *selene*, respectively [28, 66]. Present findings are consistent with the expression of the *Vg* gene at the late larval stage in lepidopteran species, e.g., *B*. *mori* [21] *A*. *pernyi* [64], and *C*. *cephalonica* [47].

The qRT-PCR results showed that of the *CcVg* gene transcript downregulation confirms the sensitivity of *C*. *cautella* toward RNAi application. Generally, the evidence that has emerged from the published data is that lepidopteran species are reported to be more tolerant to RNAi experiments when compared with other insect groups, particularly the coleopteran species, such as red flour beetles, *Tribolium castaneum* (Herbst) (Coleoptera: Tenebrionidae) [70], Colorado potato beetles, *Leptinotarsa decemlineata* (Say) (Coleoptera: Chrysomelidae) [71], and *A*. *grandis* [53]. For example, in *A*. *grandis*, a 97% reduction in the *Vg* gene expression was recorded after 72 h of Vg-based dsRNA injection [53].

The *CcVg*-based RNAi application extended the pre-oviposition periods in dsRNA-treated females, and a 50% decrease in the fecundity and hatchability assured that there was a single functional *Vg* gene in *C*. *cautella* similar to other lepidopteran species [21, 31, 47, 64, 71]. It is not always important that RNAi must affect overall ovipositional parameters, such as in the case of the *A*. *grandis*, *Vg*-based RNAi did not affect the ovipositional period and fecundity, but there was no egg hatchability [53]. By contrast, *C*. *lectularius*, egg production completely ceased within 2 weeks after *Vg*-based dsRNA injections [30].

In the present study, the peak silencing effect was recorded at 48 h post-injection, but the *CcVg* mRNA expression level started to bounce back at 72 h. The impact of dsRNA was reported to be the dose-, target gene-, and species-dependent. In *C*. *cephalonica*, adult moths injected with dsRNA of *Vg* gene showed significant downregulation of *Vg* mRNA at 24 h post-injection, whereas mRNA expression level started to recover at 72 h [47]. Similarly, the potato tuber moth, *Phthorimaea operculella* (Zeller) (Lepidoptera: Gelechiidae), third instar larvae were injected with chitin synthase enzyme A (*PhoCHSA*) dsRNA for different time intervals from 12 to 96 h, and it was observed that the climax of *PhoCHSA* transcript silencing was at 48 h post-injection and the transcript level recovered at 96 h post-injection [72]. Similar results have also been observed in *T*. *castaneum* [73].

The success of gene silencing in insect species depends on successful dsRNA delivery [52, 74, 75]. Particularly, regarding the *Vg* gene’s crucial role in insect reproduction, it has been successfully silenced in lepidopterans species [47, 74]. The key factor influencing RNAi efficiency is dsRNA uptake and its processing to siRNA at the cellular level. In the lepidopteran species, the cells and tissues are not competent enough to uptake and process the dsRNA quickly compared with those in the coleopteran species, in which the dsRNA is quickly processed into siRNA [76].

Scientists are attempting to determine possible means of dsRNA delivery either through transgenic plants or feeding of dsRNA expressed by bacteria [52, 71]. The knockdown of the *Vg* gene by RNAi might have the ability to suppress reproductive traits in *C*. *cautella*, and *CcVg* could be a promising target gene to develop a pest management tactic for *C*. *cautella*. Thus, future RNAi research should direct its attention to dsRNA delivery to manage *C*. *cautella* in field/storage conditions.

## Conclusions

The present research is a comprehensive report on molecular characterization, expression profile, and silencing of the *CcVg* gene through RNAi. In comparison with other lepidopteran insects, the *CcVg* gene structure is conserved, and the phylogenetic study showed that *CcVg* has closer ancestry with other lepidopteran species. The expression pattern revealed that *Vg* is expressed explicitly in females and began to be expressed in late female larvae; then, its expression gradually increased with the development stage and was at its peak on day one for the adult female moth. The *CcVg*-based RNAi study revealed that *CcVg* is the only primary functional gene in *C*. *cautella*. The silencing of *CcVg* up to 90% revealed the potential of emerging RNAi technology for pest management. To achieve successful results, future research should focus on the proper delivery of dsRNA.

## Supporting information

S1 Fig The PCR-amplified target region of the *CcVg* gene transcript used for RNAi experiments. The 457 bp size mentioned on the right side is the amplified *CcVg* mRNA template used to synthesize the *CcVg*-based dsRNA. The amplified band was separated on an agarose gel (1.2%) and visualized under an ultraviolet light through the BioDocAnalyze gel documentation system (Biometra). M: Molecular marker, bp: Base pair.
(TIF)

S2 Fig Sequence confirmation of the *CcVg*-based RNAi target region. Numbers on the right side are nucleotides. The T7 promoter region is in bold and underlined font at the 5ʹ end.
(TIF)

S3 Fig Quality and concentration calculation of *CcVg*-dsRNA. The concentration was measured using a NanoDrop 2000 spectrophotometer (Thermo Fisher Scientific, USA). *CcVg*-dsRNA concentration was 1089.9 ng/μL. The absorbance ratio was 2.08 at the 260/280 level, suggestive of the quality depicted on the right.
(TIF)

S4 Fig Confirmation of *CcVg*-dsRNA. Agarose gel (1.2%) was used to confirm the dsRNA. The 457 bp mentioned on the right is the synthesized *CcVg*-dsRNA. Using the BioDocAnalyze gel documentation system (Biometra), the band was visualized under ultraviolet light. M: Molecular marker, bp: Base pair.
(TIF)

S5 Fig Nucleotide and amino acid sequence of the *CcVg* cDNA. Nucleotides are numbered on the right of each line. The signal peptide is indicated by a double underline. The clusters of serine residues are in bold and underlined font. The DGQR and GL/ICG conserved motifs are present at the C-terminal and indicated with underlined font. One cleavage site (RXXR) is in bold and double-underlined font. Three possible glycosylation sites (having a consensus sequence: NXS/T) are indicated with bold font. The phosphorylated tyrosine (Y), threonine (T), and serine (S) residues are highlighted in bright yellow. Six cysteine residues are in bold and highlighted red font. The stop codon is in bold and italic font (small letters). The *CcVg* sequence was submitted to the NCBI database, and an accession number was obtained (ALN38805).
(TIFF)

S1 Table Primer used in the present study. (DOCX)

S2 Table Chemicals/Reagents, machine, and softwares used if the study. (DOCX)
